# Radiofrequency Ablation Combined with Radioactive Seed Implantation for Nonsmall Cell Lung Cancer

**DOI:** 10.1155/2022/4016081

**Published:** 2022-03-21

**Authors:** Su Chen, Zhengzuo Sheng, Naixiang Huang

**Affiliations:** Department of thoracic Surgery, FuXing Hospital, Capital Medical University, Beijing 100038, China

## Abstract

The aim of this study is to investigate the value of radiofrequency ablation combined with radioactive seed implantation in nonsmall cell lung cancer treatment. 30 patients with primary nonsmall cell lung cancer were randomly divided into two groups. Group A was treated with radiofrequency ablation combined with radiation seed implantation, and group B was treated with radiofrequency ablation only. We compared the incidence of complications in the two groups and reviewed the effective percentage every 3 months. All patients were treated successfully, and there were no deaths during treatment. There were no deaths and no cases of distant organ metastasis in nine months of follow-up. There were no significant differences in treatment-related complications between the two groups. The early postoperative (three and six months) effective percentage was not significantly different (*P* > 0.05). After 9 months, the postoperative effective rate for group A (9/15) was significantly different from that for group B (radiofrequency ablation) (6/15) (*P* < 0.05). Radiofrequency ablation combined with radiation ^125^I seed implantation can complement each other in the treatment of nonsmall cell lung cancer.

## 1. Introduction

Lung cancer is one of the most common malignant tumors in the world. According to cancer statistics, the pace of the annual decline in lung cancer mortality doubled from 3.1% during 2009 through 2013 to 5.5% during 2014 through 2018 in men, from 1.8% to 4.4% in women, and from 2.4% to 5% overall. This trend coincides with steady declines in incidence (2.2%-2.3%) but rapid gains in survival specifically for nonsmall cell lung cancer (NSCLC). In China, the incidence rate and mortality rate of lung cancer rank first among all kinds of malignant tumors. Lung cancer is a serious threat to human health, and it has become an important issue of global public health concern.

Radiofrequency ablation and radioactive ^125^I seed implantation are local lung cancer treatment methods [1–3] that have been developed in recent years. There have been many discussion about the two treatment methods at home and abroad. Thermal ablation is a new treatment for lung cancer, in which radiofrequency ablation and microwave ablation are paid more and more attention in the treatment of lung cancer. These two ablation methods are mainly used in the following two cases: one is for the curative treatment of primary lung cancer with maximum tumor diameter ≤3 cm and no metastasis and lung metastatic cancer with controlled primary focus; second, it is used for palliative treatment of primary lung cancer with tumor maximum diameter >3 cm and advanced or recurrent lung cancer after treatment by other methods.

Stereotactic body radiotherapy (SBRT) has the characteristics of single high equivalent biological dose and plays a more important role in the treatment of early NSCLC. Stereotactic radiotherapy (SBRT) uses an accurate stereotactic radiotherapy positioning system. Compared with the previous radiotherapy plans, the positioning and irradiation agents are more accurate. The normal tissues around the target area are given low-dose irradiation, and the tumor target area can implement low-dose radiotherapy. Stereotactic radiotherapy (SBRT) can give local high-dose radiotherapy to the tumor, make the local tumor achieve the ideal control effect, and minimize the toxic and side effects such as radiation reaction of normal tissue. It can effectively achieve higher local radiation dose and lower probability of complications. The application of ^125^I seeds brachytherapy (RSB) can greatly increase the local radiotherapy dose of lung cancer. Radioactive ^125^I seed implantation belongs to the field of interstitial brachytherapy and is one of the methods of radiotherapy.

In clinical practice, we found that residual and recurrent tumors have been common drawbacks of these two treatments. Based on our experience, we combined the two techniques to treat patients with nonsmall cell lung cancer, achieving good short-term local efficacy.

## 2. Materials and Methods

### 2.1. Study Patients

From August 2004 to October 2013, 30 cases of primary nonsmall cell lung cancer diagnosed and pathologically confirmed in our department of thoracic surgery were selected according to NCCN staging principles. Patients with tumors of stages I, IIA, and IIB had a KPS score over 80, median age 78 years, blood routine, biochemical routine, heart, and mostly normal lung, liver, and kidney functions. Surgery, chemotherapy, and radiotherapy were abandoned for multiple reasons (physical intolerance or subjective objections of patients and their families). The 30 patients were randomly divided into two groups of 15. There were no significant differences between groups in gender, age, and staging. The study protocol was approved by the hospital's ethical committee, the reasons for the choice of treatment and the possible situations before and after the operation were explained to the patients and their families in detail, and informed consent was obtained from all participants.

### 2.2. Equipment

Radiofrequency ablation: it was done by the RITA radiofrequency ablation system. All data in the treatment process were recorded in real time using an online computer. Radioactive therapy: ^125^I particles were provided by the Institute of Chinese Academy of Atomic Energy. They were cylindrical, 4.5 mm long, 0.8 mm in diameter, and had a 60.4-day half-life. They release 27.4–31.5 keV X-rays and 35.5 keV gamma-rays with an initial dose rate of 7.7 cGy/h and an effective irradiation distance of 1.7–2.0 cm.

### 2.3. Treatments

Group A (combination): radiofrequency ablation of lung cancer was performed using CT-guided percutaneous puncture under intravenous and local anesthesia. After ablation, radioactive seeds were implanted according to preoperative plan. Group B (radiofrequency alone): radiofrequency ablation of lung cancer was performed using percutaneous puncture under intravenous and local anesthesia.

### 2.4. Therapeutic Evaluation and Follow-Up Analysis

For the evaluation index, enhanced CT plain scans were used to judge tumor areas and volumes. The curative effect was measured by the difference in tumor size before and after operation. The whole-body condition evaluation was mainly based on the whole-body review. For therapeutic evaluation, a comprehensive review was conducted before treatment and one month, three months, six months, and nine months after treatment. Efficacy was evaluated according to the WHO criteria: complete remission (CR): all visible lesions disappeared completely and maintained for at least four weeks; partial remission (PR): the product of the two largest vertical tumor diameters decreased by more than 50% and maintained for more than four weeks; no change (SD): the product of the two largest vertical diameters of tumors decreased by less than 50%, increased less than 25%, or no new lesions appeared; and progress (PD): the product of the two largest vertical tumor diameters increased by more than 25% or new lesions appeared. The former two are valid, while the latter two are invalid.

### 2.5. Statistical Analysis

Statistical Product and Service Solutions (SPSS) 11.5 (SPSS Inc., Chicago, IL, USA) was used for statistical analysis. Counting data were tested using the *X*^2^ test, and the measurement data were tested using a *t*-test. *P* < 0.05 was considered to be statistically significant.

## 3. Results

### 3.1. Short-Term Effects

Both groups successfully completed the treatment with no mortality. Comprehensive reviews were conducted one, three, six, and nine months after therapy to evaluate short-term efficacy. In nine months after therapy, there were no cases of distant organ metastasis. Three months after therapy, the effective rate for group A (radiofrequency ablation + radioactive seed implantation group) (12/15) was not significantly higher than for group 1 (radiofrequency ablation group) (11/15), and the difference was not significant (*P*=0.665, *P* > 0.05). There was no significant difference between groups (13/15 and 10/15, respectively) at six months (*P*=0.195, *P* > 0.05). At nine months after therapy, however, the effective rate for group A was significantly higher than that for group B (9/15 vs. 6/15, respectively) (*P*=0.0463, *P* < 0.05) (Figures 1 and 2).

### 3.2. Treatment-Related Complications

Pneumothorax: all cases had localized pneumothorax. Only three patients were treated with thoracic puncture. All other patients recovered spontaneously. There was no significant difference between groups (Figure 3).

Hemoptysis or pleural hemorrhage: there were few hemoptysis patients, all of with blood in their sputum. They improved after symptomatic treatment of hemostasis. There was no significant difference between groups. No patients with intrathoracic hemorrhage were found (Figure 3).

Fever: after radiofrequency ablation, patients developed fever that was usually about 38°C. After symptomatic treatment, patients recovered to normal within a week. There was no significant difference between groups (Figure 3). Other complications were sporadic, including pleural effusion (nonhemorrhagic) and without statistical significance.

## 4. Discussion

Radiofrequency ablation (RFA) uses electrodes to emit radiowaves to excite polar molecules in the surrounding tissues, causing high-speed oscillation, colliding, and friction with adjacent molecules [4]. This process converts radiofrequency energy into heat energy. Dupuy et al. first reported three cases of lung cancer treated with RFA in 2000; since then, it has been widely used to treat lung cancer.

In our clinical work, we found that tumor shrinkage was not obvious after radiofrequency ablation in many patients, so we used lung biopsy and pathological evaluation. Comparisons before and after ablation showed that residual tumors were the primary reason for its poor efficacy.

One shortcoming of radiofrequency ablation is a heat sink effect, in which rapid blood flow in the tumor area takes away part of the heat generated by RFA. This has been termed the “heat drop effect,” which can lead to the incomplete treatment of tumors near large vessels and the trachea and cause tumor recurrence. When the tumor is large or irregular in shape, it also is likely to result in residual tumors and recurrence. Another issue is that the lung is a gas-containing organ wrapping tumors. Therefore, some of the heat generated by RFA can easily be carried away by gas, reducing temperatures at the edges of tumors. These shortcomings explain why the efficacy of radiofrequency ablation for lung cancer is obviously worse than it is for tumors in other tissues [5–7].

Implantation of radioactive particles is a relatively new treatment for lung cancer. It has the advantage of increased energy release. It can be provided continuously because it causes little or no damage to surrounding normal tissues, reducing proliferation. It has been shown that the doubling time of nonsmall cell lung cancer (adenocarcinoma or squamous cell carcinoma) cells is 15–17 days, with ^125^I reducing doubling time to more than 10 days [8–10].

Radiofrequency ablation combined with radioactive seed implantation has been widely used to treat malignant tumors in other organs, including the liver, pancreas, and nasopharynx [11–13].

Our data suggest that the combination of radiofrequency ablation plus radioactive seed implantation is superior, at least in short-term. The effects of radiofrequency ablation appear early, and the local condition of patients is relieved soon after therapy. However, residual tumor soon begins to grow, so the therapeutic effect cannot be consolidated. In contrast, the therapeutic effect of radioparticle implantation is much slower, requiring more than two months to appear. Since the distance over which radioparticle therapy acts is shorter, the tumor is not significantly reduced after 2-3 half-lives in most patients. Radiofrequency ablation and radioactive seed implantation are therefore complimentary and maintain the effect of local treatment to the greatest extent. The long-term survival rate and metastasis-free survival rate in group A were significantly better than in group B [14–16].

In this study, we observed few complications with the treatment. Fever is more common after radiofrequency ablation, but it generally resolves within a week. Hemoptysis (including intrathoracic hemorrhage) and pneumothorax were rare, with no significant difference between groups. Most importantly, combining treatments did not significantly increase the incidence of complications.

The limitation of this study is that the number of patients in the group is still small, which may have limited application to the whole clinical in statistics, but it also gives a new clinical idea of treatment. In addition, the follow-up time is not long enough. If the follow-up time is longer, more clinical results will be obtained. In addition, this study is a single center study. If it is a multicenter joint study, it has more clinical significance. It should be noted that all the patients selected here were early stage patients. This choice was made to exclude the influence of changes in patients' general condition caused by multiple metastases. However, in the clinic, radiofrequency ablation combined with radioactive particles for the local treatment of advanced lung cancer is still effective and can be used as a part of comprehensive lung cancer treatment in clinical practice.

## 5. Conclusions

In conclusion, radiofrequency ablation combined with radioactive ^125^I seed implantation in the treatment of nonsmall cell lung cancer can achieve synergistic advantages. It achieved relatively good local short-term efficacy and is therefore worthy of further research and promotion.

## Figures and Tables

**Figure 1:** H&E staining for the tissues at different time points. (a) H&E staining of tissues before radiofrequency ablation (magnification: 10 × 5). (b) H&E staining of tissues from biopsy immediately after radiofrequency ablation (magnification: 10 × 5).

**Figure 2:** Pulmonary CT images before and after treatment. (a) Preoperative manifestations of right upper lobe lung cancer. (b) CT-guided radiofrequency ablation. (c) Three months after operation, CT scan was performed and puncture biopsy was performed to confirm the residual tumors.

**Figure 3:** Pulmonary CT images before and after treatment. (a) Radiofrequency ablation was performed for right lower lobe peripheral lung cancer. Radioactive particle implantation was performed immediately after operation. (b) At 3 months after operation, a small amount of tissue necrosis and void formation observed in the ablation and implantation areas. (c) Six months after operation, the tumor necrosis was obvious, forming a large cavity, and the treatment effect was remarkable.

## Data Availability

The datasets used and analyzed during the current study are available from the corresponding author upon request.
